The article "LncRNA OIP5-AS1 Knockdown Facilitated the Ferroptosis and Immune Evasion by Modulating the GPX4 in Oesophageal Carcinoma" was retracted in 2023. Reasons: unreliable results or conclusions; lack of ethics approval or compliance; concerns about the data; concerns about the peer review.

# LncRNA OIP5-AS1 Knockdown Facilitated the Ferroptosis and Immune Evasion by Modulating the GPX4 in Oesophageal Carcinoma

**DOI:** 10.1155/2022/8103198

**Published:** 2022-07-15

**Authors:** Junyi Hou, Qin Huang, Zhengyang Fan, Hongyang Sang, Song Wu, Shaofeng Cheng, Qianping Li

**Affiliations:** ^1^Department of Gastroenterology, Shanghai Jiao Tong University Affiliated Sixth People's Hospital, 200233, China; ^2^Department of Pathology, Shanghai Jiao Tong University Affiliated Sixth People's Hospital, 200233, China; ^3^Department of Cardiothoracic Surgery, Shanghai Jiao Tong University Affiliated Sixth People's Hospital, 200233, China

## Abstract

**Objective:**

Oesophageal cancer (EC) is an extremely invasive malignancy, which has bad prognosis that requires safe and effective treatment modalities. Immunotherapy has provided new ideas for the treatment of EC in recent years. This project was conducted to probe into the role and mechanism of lncRNA OIP5-AS1 in ferroptosis and immunotherapy of EC.

**Methods:**

Cell viability and multiplication were assessed through CCK-8, colony formation assays. Levels of Fe^2+^, MDA, and lipid ROS were applied to determine ferroptosis. GPX4 and OIP5-AS1 levels were examined through real-time PCR assay. The relationship between OIP5-AS1 and GPX4 was estimated through RNA immunoprecipitation assay. Flow cytometry was applied to examine the effect of OIP5-AS1 on CD8+ T cells.

**Results:**

OIP5-AS1 inhibition significantly inhibited EC cell viability and proliferation, induced ferroptosis, and downregulated GPX4 levels, while GPX4 reversed these effects. OIP5-AS1/GPX4 induced CD8+ T cell interaction and induced apoptosis through PD-1/PD-L1 immune checkpoints of CD8+ T cells.

**Conclusion:**

OIP5-AS1/GPX4 promotes EC development and relieved ferroptosis; furthermore, OIP5-AS1/GPX4 facilitated immune evasion via modulation of PD-1/PD-L1, suggesting aiming at OIP5-AS1 is a possible route which might enhance the effectiveness of immunotherapy.

## 1. Introduction

Oesophageal carcinoma (EC) acts as a malignant tumour, which occurs in the squamous or glandular epithelium of the oesophagus, and it is familiar in human cancers, occupying over 90% of oesophageal tumours, the incidence of which is increasing worldwide [1]. Despite improvements in available therapies, due to local infiltration and distant metastases, overall survival probability of sufferers with oesophageal cancer remains disappointed [2]. In a number of tumour suppressors and in the proceeding and development of EC, oncogenes have been confirmed to do a vital part [3], whereas in the carcinogenesis and progression of EC, the exact molecular mechanisms remain to be entirely expounded. Therefore, understanding the molecular mechanisms of EC will provide guidance for the treatment, screening, and early detection of oesophageal cancer.

The article "LncRNA OIP5-AS1 Knockdown Facilitated the Ferroptosis and Immune Evasion by Modulating the GPX4 in Oesophageal Carcinoma" was retracted in 2023. Reasons: unreliable results or conclusions; lack of ethics approval or compliance; concerns about the data; concerns about the peer review.

Although the standard treatment options for EC are varied [4], the prognosis for patients with oesophageal cancer is still poor [5]. Immunotherapy has provided new treatment ideas for a variety of malignancies and has greatly relieved malignant melanoma, nonsmall cell lung cancer, liver cancer, and other tumours, and it improves the survival possibility of patients [6]. Many clinical trials have confirmed that immunotherapy combined with radiotherapy can enhance the antitumour effect of stage II and III patients [7]. Tumour immunotherapy targeting immune checkpoints is now a new hope for EC treatment [8]. Among the many immune checkpoint signaling factors, programmed death protein-1/programmed death protein-1 ligand (PD-1/PD-L1) plays an important role in the tumour immune process, inducing a tumour immunosuppressive microenvironment and promoting tumour proliferation and metastasis [9]. A study shows that high PD-L1 level is greatly related to survival rates in tumour patients [10], aiming at PD-1/PD-L1 is concerned with clinical prognosis.

Long noncoding RNAs (lncRNAs) are not only important regulators of normal cell growth, differentiation, apoptosis, and tissue metabolism but also do a part in the proceeding of many diseases, and lncRNAs have become potential targets for disease therapy [11]. OPA-interacting protein 5 antisense transcript 1 (OIP5-AS1) is localized on chromosome 15q15.1, is well conserved during vertebrate evolution, and is involved in cancer progression [12]. A previous study has suggested that OIP5-AS1 regulates tumour progression as an oncogenic or pro-oncogenic gene [13]. A previous study has suggested that OIP5-AS1 promotes proliferation and metastasis of EC cells [14]. Furthermore, a research shows that OIP5-AS1 inhibits ferroptosis and promotes cancer progression in prostate cancer [15], whereas the importance needs to be further investigated of OIP5-AS1 in EC. In view of the above research basis, the regulation of OIP5-AS1 in EC cell ferroptosis and activity, as well as the regulation of immunotherapy, was explored in this study, and also the molecular mechanism of OIP5-AS1 action was explored, with a view to providing new ideas for the treatment of EC.

## 2. Materials and Methods

### 2.1. Cell Culture and Transfection

Human oesophageal cancer cell lines Eca109, TE-13, TE-1, and TTN and normal oesophageal epithelial cell line HEEC were bought from Shanghai Bogu Biotechnology Co. Cells were cultivated in a sterile incubating device under 37°C, 5% CO_2_, and 5% v/v. The pcDNA3.1-OIP5-AS1/si-OIP5-AS1 vector plasmid and its negative control were constructed by GenePharma (Shanghai, China). Blank plasmids were used as controls. EC cells at logarithm growth phase were inoculated in 6-well dishes and transfected with control and pcDNA3.1-OIP5-AS1/si-OIP5-AS1 at 70%-80% cell fusion through the instructions of Lipofectamine 2000 (Invitrogen; ThermoFisherScientific, Inc.). After 48 h of transfection, all RNA was gotten and qRT-PCR was conducted to demonstrate the efficiency of transfection.

The article "LncRNA OIP5-AS1 Knockdown Facilitated the Ferroptosis and Immune Evasion by Modulating the GPX4 in Oesophageal Carcinoma" was retracted in 2023. Reasons: unreliable results or conclusions; lack of ethics approval or compliance; concerns about the data; concerns about the peer review.

### 2.2. CCK-8 Assay

The cells were made into a single-cell suspension and counted. After the cells were attached to the wall, each plate was removed and 10 *μ*L of CCK-8 reagent (Sigma, USA) was added to each well to measure the absorbance at different time points (24 h, 48 h, 72 h, 96 h). The absorbance (A) of each well was measured at 450 nm wavelength on an enzyme marker and repeated three times to obtain the average value.

### 2.3. QRT-PCR

The transfected hBMSCs were collected, all RNA was gotten from the samples by TRIzol method, RNA concentration was determined spectrophotometrically, and cDNA was synthesized by reverse transcription. QRT-PCR was performed according to SYBRPremix ExTaqTM II kit instructions (TaKaTa, Japan). Reaction conditions: 95°C, 0.5 min; 95°C, 5 s, 58°C, 0.5 min, 40 cycles; 95°C, 15 s, 58°C, 0.5 min, 95°C, 15 s. Using GAPDH as internal reference, the 2^-*ΔΔ*Ct^ way was utilized to get miR-103-3p, OIP5-AS1, and GPX4 levels. All primer sequences were synthesized by Guangzhou Ribo Bio (China).

### 2.4. Plate Clone Formation Assay

Cells were taken at logarithmic growth stage, digested routinely, and single-cell suspensions were prepared and counted. Cells were inoculated in a 6-well plate at 1000 cells/2 mL/well; the dish was gently shaken in a cross direction to disperse the cells and incubated routinely at 37°C in 5% CO_2_ for 10~14 d. When clones were visible to the naked eye in the dish, the culture was terminated; the culture fluid was discarded, washed twice with PBS, and air dried. Methanol was fixed for 15 min, discarded, and air dried. Stained with Gimsa stain for 10 min, washed off the stain slowly under running water, air dried, photographed, and counted.

### 2.5. Western Blot

The transfected cells were lysed and protein extracted, protein content was measured, the volume of the upper sample was determined, and 10% polyacrylamide gel was developed according to the size of Ki67 and PCN1 molecular weight; anhydrous ethanol was used to close the separation gel, anhydrous ethanol was poured off after 40 min, ultrapure water was washed 3 times, with concentrated gel inserted into the comb, and electrophoresis was started after 30 min of polymerization. After completion of electrophoresis, the gel was removed and dipped into the transfer solution, PVDF membrane was transferred and closed for 1 h, then diluted primary antibody (1 : 800) was added and incubated overnight at 4°C on a shaker. The strips were removed the next day, washed 3 times in TBST, placed in a centrifuge tube and incubated with secondary antibody for 1 h at room temperature, and washed 3 times in TBST. ECL detection reagent was prepared, dropped onto PVDF membrane, reacted for 1 ~ 2 min, and tested on the machine and the results were analyzed.

The article "LncRNA OIP5-AS1 Knockdown Facilitated the Ferroptosis and Immune Evasion by Modulating the GPX4 in Oesophageal Carcinoma" was retracted in 2023. Reasons: unreliable results or conclusions; lack of ethics approval or compliance; concerns about the data; concerns about the peer review.

### 2.6. RNA Immunoprecipitation Assay

RNA immunoprecipitation was acted according to the Magna RIP RNA-binding protein immunoprecipitation. The experiments were performed according to the instructions of the Magna RIP RNA-binding protein immunoprecipitation kit (Millipore, Germany), with the addition of AGO2 and IgG antibodies added to the protein precipitates, and the target RNA was detected by PCR. The target RNA expression in the precipitates was detected by PCR.

### 2.7. Flow Cytometry

The cells were inoculated in 96-well plates at 1 × 10^4^ cells/well, incubated for 24 h, cleaned twice in PBS, subjected to fixation in 70% ethyl alcohol, and obtained all the night under 4°C. Cells were cleaned once in PBS and the cellular density was changed to 1 × 10^6^ cells/mL. Propidium iodide dyeing liquor was put to an eventual content of 0.05 mg/mL and stained for 30 min at 4°C. All groups were analyzed by flow cell technique. The cellular cycle was analyzed by flow cell technique. Three replicate wells were set up for all groups, and the similar test was made three times and the mean result was taken.

### 2.8. Statistical Analysis

According to SPSS 22.0 statistical program (America), statistic assay was completed. Measures were shown as average ± SD (*x* ± *s*), *t*-test was utilized to make a comparison of sample means between groups, one-way ANOVA was utilized for comparing several sample means, and SNK-q test was used for two-way comparison.

## 3. Results

### 3.1. OIP5-AS1 Inhibited Ferroptosis and Promoted EC Progression

Erastin and RSL3 are extensively used to be ferroptosis stimulator [16]. OIP5-AS1 significantly relieved Erastin and RSL3-exposed inhibition of cell vitality as shown in Figures 1(a) and 1(b). Later on, the markers of ferroptosis, including the enhanced levels of Fe^2+^, MDA, and lipid ROS (*p* < 0.05, Figures 1(c)–1(e)), were notably inhibited by OIP5-AS1, suggesting the inhibition of ferroptosis. In subsequence, vitality and multiplication of EC cells were examined caused by OIP5-AS1. Firstly, in all four EC cell lines, the OIP5-AS1 level was upregulated (*p* < 0.05, Figure 1(f)). Comparing with OIP5-AS1 negative control, OIP5-AS1 notably accelerated cell proliferation curve (*p* < 0.05, Figure 1(g)), as well as colony formation ability (*p* < 0.05, Figure 1(h)).

The article "LncRNA OIP5-AS1 Knockdown Facilitated the Ferroptosis and Immune Evasion by Modulating the GPX4 in Oesophageal Carcinoma" was retracted in 2023. Reasons: unreliable results or conclusions; lack of ethics approval or compliance; concerns about the data; concerns about the peer review.

### 3.2. OIP5-AS1 Knockdown Promoted Ferroptosis and Inhibited the Progression of EC

Later on, in EC, the impact of OIP5-AS1 was estimated ulteriorly by transfecting si-OIP5-AS1 to construct OIP5-AS1 low-expressing EC cell lines. Erastin and RSL3-exposed inhibition of cell vitality was substantially exacerbated by si-OIP5-AS1 (*p* < 0.05, Figures 2(a) and 2(b)). Besides, the markers of ferroptosis, including the enhanced levels of Fe^2+^, MDA, and lipid ROS (*p* < 0.05, Figures 2(c)–2(e)), were particularly strengthened by si-OIP5-AS1, indicating the occurrence of ferroptosis. In subsequence, comparing with OIP5-AS1 negative control, si-OIP5-AS1 notably suppressed cell proliferation curve (*p* < 0.05, Figure 2(f)), As well as colony formation ability (*p* < 0.05, Figure 2(g)).

### 3.3. OIP5-AS1 Interacted with GPX4 in EC Cells

Furthermore, RNA immunoprecipitation results showed that OIP5-AS1 enriched more GPX4 mRNA compared to the lgG group (*p* < 0.05, Figure 3(a)). The results showed that GPX4 inhibited by si-OIP5-AS1 was promoted by GPX4 (*p* < 0.05, Figure 3(b)) and that GPX4 significantly attenuated the inhibition of cell viability induced by Erastin and RSL3 compared to the si-OIP5-AS1 group (*p* < 0.05, Figures 3(c) and 3(d)). GPX4 significantly inhibited si-OIP5-AS1-induced ferroptosis, including a decrease in Fe^2+^, MDA, and lipid ROS levels (*p* < 0.05, Figures 3(e) and 3(g). Subsequently, GPX4 significantly increased the cell proliferation profile compared to the si-OIP5-AS1 group (*p* < 0.05, Figure 3(h)). Colony formation was enhanced (*p* < 0.05, Figure 3(i)).

### 3.4. Via PD-1/PD-L1 Immune Checkpoint, OIP5-AS1 Induced Apoptosis of CD8+ T Cells

Tumour cells interact with CD8+ T cells, which have been reported in the tumour microenvironment and interfere with their cytotoxic function [17]. Therefore, we hypothesized that CD8+ T cells could be altered via OIP5-AS1/GPX4 in EC. Later on, EC cells were co-cultured with CD8+ T cells, in order to imitate the tumour microenvironment. In CD8+ T cells, an upregulation in the percentage and a decrease in apoptosis were showed by flow cytometry analysis, whereas a reversal of GPX4 in the presence of OIP5-AS1 knockdown (*p* < 0.05, Figures 4(a) and 4(b)). In addition, as PD-1/PD-L1 interaction inhibits CD8+ T cell activity and enhances immune evasion in tumours [18], we hypothesized that via the PD-1/PD-L1 checkpoint OIP5-AS1/GPX4 could regulate CD8 + T cell alterations (*p* < 0.05, Figures 4(c) and 4(d)). In subsequence, in a co-culture system, antibodies opposing PD-1 and PD-L1 were adopted to block PD-1/PD-L1 in order to affirm our hypothesis. Thus, in TTN and TE-13 cells, OIP5-AS1 and GPX4 declined the CD8+ T cells proportion, meanwhile strengthened CD8 + T cells apoptosis, and anti-PD-1 or anti-PD-L1 treatment could reverse this condition (*p* < 0.05, Figures 4(e) and 4(f)). In a word, OIP5-AS1/GPX4 together induced EC cell-CD8+ T cell interactions and triggered CD8+ T cell apoptosis via PD-1/PD-L1 immune checkpoints.

The article "LncRNA OIP5-AS1 Knockdown Facilitated the Ferroptosis and Immune Evasion by Modulating the GPX4 in Oesophageal Carcinoma" was retracted in 2023. Reasons: unreliable results or conclusions; lack of ethics approval or compliance; concerns about the data; concerns about the peer review.

## 4. Discussion

EC is one of the common malignancies of the upper gastrointestinal system and is currently ranked as the 8th most common cancer in the world [19]. In China, oesophageal cancer ranks 5^th^ in incidence of malignant tumours, with 287,000 new cases and 211,000 deaths per year, predominantly in men [20]. The early symptoms of oesophageal cancer are not obvious, and most patients present with clinical symptoms such as dysphagia and seek medical consultation, at which time the disease is mostly at an advanced stage, which is the main factor for the poor prognosis and low survival rate of oesophageal cancer [21]. As a class of molecular markers closely related to tumours, lncRNAs play an important role in the development and progression of EC. In the current study, we found that OIP5-AS1 was closely associated with the development of EC Figure 5.

A previous study suggests that OIP5-AS1 can promote EC progression by targeting miR-1297 [22]. Similarly, OIP5-AS1 expression is upregulated in EC tissues and cells and is able to promote EC progression by regulating miR-30-5p [14]. In line with the above studies, in the current study, we found that OIP5-AS1 expression was upregulated in EC cells and that OIP5-AS1 was able to inhibit the proliferation of EC cells. Glutathione peroxidase (GPX) is a collective term for a group of peroxidases widely found in animals, and GPX4 is one of the most important members of this enzyme family. Lee et al. have found that GPX4 overexpression is associated with local lymph node metastasis and clinical staging in oral squamous cell carcinoma [23]. Overexpression of GPX4 in human hepatocellular carcinoma, compared to controls, may play a role in higher tumour grade [24]. Furthermore, the study suggests that GPX4 promotes EC progression [25]. In the current study, we confirmed the binding of OIP5-AS1 to GPX4 by RNA immunoprecipitation assays, in addition confirmed that OIP5-AS1 knockdown was able to inhibit EC cell proliferation by downregulating GPX4.

Currently, apoptosis, necrosis, pyroptosis, and ferroptosis have been identified. Ferroptosis is accompanied by a significant increase in intracellular iron ion flow, reactive oxygen species (ROS), and lipid peroxidation levels, culminating in membrane breakdown and cell death due to lipid peroxidation of the phospholipid lining of the cell membrane [26]. However, there is considerable evidence that GPX4 can be used as a reference marker for determining cellular ferroptosis [27]. Inactivation of GPX4 protein, which has the function of scavenging lipid peroxides, leads to disruption of oxidative homeostasis and disruption of membrane structure by lipid peroxides, triggering ferroptosis [28]. Fe^2^^+^, MDA, and lipid ROS as key markers of ferroptosis [29]. In the current study, we found that si-OIP5-AS1 significantly promoted Fe^2+^, MDA, and lipid ROS, suggesting that OIP5-AS1 inhibits ferroptosis, and furthermore, we found that GPX4 alleviated the ferroptosis-promoting effect of si-OIP5-AS1.

The article "LncRNA OIP5-AS1 Knockdown Facilitated the Ferroptosis and Immune Evasion by Modulating the GPX4 in Oesophageal Carcinoma" was retracted in 2023. Reasons: unreliable results or conclusions; lack of ethics approval or compliance; concerns about the data; concerns about the peer review.

Tumour-induced immunosuppression is one of the main mechanisms by which tumours proliferate and evade the immune system. Tumour cells use multiple immunosuppressive pathways to resist tumour immunity, one of which is through the PD-1/PDL1 axis, which is an important “immune checkpoint” [30]. The PD-1/PD-L1 pathway plays a key role in chronic infection, tumour immune escape, and the formation of the tumour microenvironment [31]. PD-L1 causes T-cell depletion and immune tolerance and is thought to be a major contributor to tumour immune escape [32]. In addition to being widely expressed on the surface of T lymphocytes, B lymphocytes, dendritic cells, and macrophages, PD-L1 is also found to be highly expressed on the surface of many tumour cells. Thus, a variety of cytokines and exosomes in the tumour microenvironment can induce PD-L1 expression and enhance PD-1/PD-L1 signaling to inhibit the activation of cytotoxic T lymphocytes in the tumour microenvironment, thereby promoting tumour escape [33]. In the current study, we applied antibodies against PD-1 and PD-L1 to block PD-1/PD-L1 in a co-culture system. Consequently, in TTN and TE-13 cells, OIP5-AS1 and GPX4 reduced the proportion of CD8+ T cells and promoted apoptosis of CD8+ T cells, a phenomenon that could be reversed by anti-PD-1 or anti-PD-L1 treatment. This suggests that OIP5-AS1/GPX4 together induces EC cell-CD8+ T cell interaction and triggers CD8+ T cell apoptosis via PD-1/PD-L1 immune checkpoints.

However, the present study has some limitations and the study of OIP5-AS1 in EC clinical samples needs to be further explored, in addition whether OIP5-AS1 acts other targets in EC cell ferroptosis and immunotherapy needs to be investigated. In summary, OIP5-AS1 knockdown promotes ferroptosis and immune evasion in oesophageal cancer through regulation of GPX4, and OIP5-AS1 may serve as a clinical prognostic marker in ferroptosis-based cancer research and immunotherapy.

The article "LncRNA OIP5-AS1 Knockdown Facilitated the Ferroptosis and Immune Evasion by Modulating the GPX4 in Oesophageal Carcinoma" was retracted in 2023. Reasons: unreliable results or conclusions; lack of ethics approval or compliance; concerns about the data; concerns about the peer review.

## Figures and Tables

**Figure 1:** OIP5-AS1 inhibited ferroptosis and promoted EC progression. (a, b) OIP5-AS1 regulated the inhibitory effect of Erastin and RSL3 on cell viability. (c–e) Markers of ferroptosis, including the enhanced levels of Fe2+, MDA, and lipid ROS. (f) In all four EC cell lines, the OIP5-AS1 level was detected by QRT-PCR. (g, h) CCK-8 and colony formation were applied to assess EC cell viability. ∗*p* < 0.05, ∗∗*p* < 0.01, ∗∗∗*p* < 0.001. All experiments were repeated three times.

**Figure 2:** OIP5-AS1 knockdown promoted ferroptosis and inhibited the progression of EC. (a, b) si-OIP5-AS1 regulated the inhibitory effect of Erastin and RSL3 on cell viability. (c–e) Markers of ferroptosis, including the enhanced levels of Fe2+, MDA, and lipid ROS. (f, g) CCK-8 and colony formation were applied to assess EC cell viability. ∗*p* < 0.05, ∗∗*p* < 0.01, ∗∗∗*p* < 0.001. All experiments were repeated three times.

**Figure 3:** OIP5-AS1 interacted with GPX4 in EC cells. (a) RNA immunoprecipitation was used to detect their interaction. (b) GPx4 was detected by qRT-PCR. (c, d) si-OIP5-AS1 regulated the inhibitory effect of Erastin and RSL3 on cell viability. (e–g) Markers of ferroptosis, including the enhanced levels of Fe^2+^, MDA, and lipid ROS. (h, i) CCK-8 and colony formation were applied to assess EC cell viability. ∗*p* < 0.05, ∗∗*p* < 0.01, ∗∗∗*p* < 0.001. All experiments were repeated three times.

**Figure 4:** Via PD-1/PD-L1 immune checkpoint, OIP5-AS1 induced apoptosis of CD8+ T cells. (a, b) Percentage and apoptosis of CD8+ T cells were showed by flow cytometry analysis. In a co-culture system, antibodies opposing PD-1 and PD-L1 were adopted to block PD-1/PD-L1. (a, b) Percentage and apoptosis of CD8+ T cells were showed by flow cytometry analysis in EC cells. ∗∗*p* < 0.01, ∗∗∗*p* < 0.001. All experiments were repeated three times.

**Figure 5:** OIP5-AS1 knockdown promoted ferroptosis and immune evasion in oesophageal cancer through regulation of GPX4.

## Data Availability

No data were used to support this study.
